The article "Cross-Border Supply Chain System Constructed by Complex Computer Blockchain for International Cooperation" was retracted in 2023. Reasons: unreliable results or conclusions; concerns about the data; concerns about the peer review; concerns about the citations.

# Cross-Border Supply Chain System Constructed by Complex Computer Blockchain for International Cooperation

**DOI:** 10.1155/2022/6221211

**Published:** 2022-04-11

**Authors:** Xiaoguang Deng, Yuxuan Ouyang

**Affiliations:** ^1^Economics and Management School, Wuhan University, Wuhan 430072, Hubei, China; ^2^Columbia University, New York, NY 10027, USA

## Abstract

The rapid development of China's local e-commerce and the continuous improvement of its business model have not only pushed the country to the forefront of the globe but also opened up the unprecedented potential for China's cross-border e-commerce. Therefore, it is imperative to build a balanced and sustainable cross-border e-commerce system, and cross-border e-commerce on the Silk Road has become a new highlight of China's e-commerce development. This study proposes a cross-border supply chain model based on the complex computer blockchain for international cooperation scenarios, contrasts and analyzes decision making in two cross-border supply chain scenarios with and without blockchain implementation, and investigates the sufficient conditions for blockchain implementation in the cross-border supply chain from the perspective of various value objectives. The analysis reveals that the cross-border supply chain has sufficient incentive to implement blockchain when the value gain generated by implementing blockchain is high or the value gain is low but the potential market size weakening factor of cross-border products is greater than a certain degree. It demonstrates that the link between cross-border product price elasticity, manufacturer cross-border effort cost, and customer cross-border preference degree would impact the circumstances for adopting blockchain in cross-border supply chains. The model also lays out a plan for the government to improve cross-border e-commerce logistics, strengthen oversight, and create a regional financial service network system to reduce credit risk.4

## 1. Introduction

The core concept of the Belt and Road initiative is to support energy and infrastructural development in Central Asia, Southeast Asia, Eastern Europe, and other associated nations in the area, as well as economic growth in these countries [1]. Similarly, the One Belt, One Road initiative has yielded positive results and created favorable conditions for the growth of cross-border e-commerce in China [2].

Cross-border e-commerce continues to expand and strengthen the collaboration between countries. With the global integration of the economy and the rapid development of Internet technology, cross-border e-commerce is developing rapidly and has become an effective strategy to promote economic growth in various economies. Cross-border e-commerce is a mode of realizing people's consumption needs by sending goods by mail between nations using the Internet as the backbone. [3]. The existence of complementary and similar consumption structures among the countries along the Belt and Road has made cross-border e-commerce extremely viable since its birth.

At this point, economic and trade exchanges between “Belt and Road” nations are increasing, trade cooperation is developing, cross-border e-commerce is growing rapidly, and collaboration is intensifying [4]. Currently, China's transactions with nations like Cambodia, Kuwait, the United Arab Emirates, and Austria increased by more than 100%, indicating that commodities from the “Belt and Road” continue to be embraced by Chinese customers. Meanwhile, by the end of 2019, China developed e-commerce cooperation structures with 22 nations, as well as deep and effective policy communication and industry engagement. [5]. Cross-border e-commerce cooperation among countries along the Silk Road has gradually increased in areas such as electricity, railroads, and finance, and cooperation among countries along the Silk Road has further deepened [6].

The development of cross-border e-commerce is inseparable from the support of the supply chain, which is a network chain structure jointly constructed by the core enterprises and consumers involved in the process of commodity circulation. As shown in Figure 1, the cross-border supply chain is a typical complex distributed scenario, which not only involves many types of role entities such as suppliers, customers, distributors, and consumers, but also contains a variety of data such as goods flow, capital flow, and information flow [7]. It can be observed that integrating the complicated data flow, sharing data securely across different players that do not completely trust each other, and promoting secure collaboration among multiple stakeholders in the supply chain are the key to improving overall supply chain efficiency. Location technology is naturally suitable for solving the above-mentioned supply chain industry problems [8].

The block supply chain is a supply chain system based on blockchain which helps in building a trusted supply chain alliance based on the blockchain network to share data securely. The blockchain data structure is used to achieve accurate traceability of supply chain data, ensuring that each link of data can be confirmed through the quality of digital signature and time-stamped proof of existence. It can effectively solve disputes between participating entities in the supply chain, realizing easy evidence and establishing rights and responsibilities [9]. Although blockchain technology has effectively solved the problem of lack of trust among supply chain entities, it has also introduced new problems. On the one hand, the redundant storage nature of blockchain technology brings great disk space consumption, causing considerable storage pressure on the server. On the other hand, the current blockchain applications present multidimensional heterogeneity, which differs in the choice of the underlying platform and business logic design [10, 11].

This study proposes a model of cross-border supply chain system based on complex computer blockchain for international economic cooperation scenarios, compares and analyzes the decision making in two scenarios of unimplemented and implemented blockchain in the cross-border supply chain, and explores the sufficient conditions for implementing blockchain in the cross-border supply chain from the perspective of different value objectives. Furthermore, the present analysis reveals that the relationship between the price elasticity coefficient of cross-border products, the cross-border effort cost coefficient of manufacturers, and the cross-border preference degree of consumers will influence the conditions for implementing blockchain in cross-border supply chain.

The rest of the manuscript is structured as follows: Section 2 is about related works. In Section 3, the proposed model is described, and different assumptions are illustrated.  Section 4 illustrates the cross-border supply chain.  Section 5 provides an analysis of blockchain implementation conditions under different value objectives.  Section 6 explains the different results, and Section 7 concludes the manuscript.

## 2. Related Work

Cross-border e-commerce is a type of business activity in which the main body of the transaction is transactions between different customers, and the two sides reach an agreement through the e-commerce platform to complete the transaction by carrying out payment and settlement and transporting goods across the border. The circulation of products has slowed in recent years as the global economy's and trade's growth rates have slowed. To address this issue, the flow of goods must be increased continuously, and the economy's and trade's growth rates must be boosted. More and more businesses are reducing the gap between themselves and international consumers to increase commodities sales. Cross-border e-commerce should be shipped out in this economic climate; now, cross-border e-commerce is still increasing swiftly, progressively altering the global economic trend.

In recent years, along with the rapid development of cross-border e-commerce and blockchain technology, more and more experts, scholars, and business people are committed to exploring the innovation and application implementation of the block supply chain. Chen [12] proposed a blockchain-based dynamic multicenter collaborative authentication model for supply chains, introduced a blockchain transaction structure applicable to fusing business-to-business (B2B) and business-to-customer (B2C) supply chain electronic transactions, and analyzed the problems faced by the diffusion of blockchain technology in B2B + B2C supply chains. The blockchain transaction structure for electronic transactions in supply chains integrating B2C models was introduced, and the problems faced in promoting blockchain technology in B2B + B2C supply chains were analyzed. Iyama et al. [13] constructed a blockchain e-commerce product traceability and anti-counterfeiting model, using blockchain technology to trace product information and prevent tampering. The authors in [14] proposed a scheme combining blockchain, Bitcoin protocol deterministic hierarchical wallet, and multiple signature technologies to meet the needs of product coding, authority management, transfer of physical rights, product traceability, and anti-counterfeiting verification in the supply chain. Cheung et al. [15] applied blockchain to the medical supply chain, using federated chain technology combined with ethereal smart contracts and encrypted Quick Response (QR) codes to record data of each transportation link and ensure authenticity and reliability of drug transportation information. Blockchain technology was used in [16] to enhance the resilience of the supply chain and analyze various risks faced by the current supply chain, and the specific application scenarios of blockchain technology in the supply chain were described. Almaktoom et al. [17] designed an authentication protocol based on the blockchain and RFID for the supply chain in the 5G mobile edge computing environment to better trade-off the overhead of supply chain communication between security and computational cost and improve the security of supply chain information transmission.

Tencent (Tencent Holdings Ltd., China) has signed a strategic cooperation agreement with China Federation of Logistics and Purchasing to launch a block supply chain alliance and waybill platform. Jingdong (Chinese e-commerce company, Beijing) released a blockchain anti-counterfeiting traceability open platform, which is free and open to brands within the Jingdong ecology [18]. Huawei (Huawei Technologies Co.) launched a blockchain service (BCS) in Huawei Cloud and described the application scenarios of blockchain technology in the supply chain field. Walmart first collaborated with IBM to design a trusted food solution based on the super ledger blockchain system, which is based on IBM's blockchain system, to transport fresh products and achieve real-time, end-to-end product traceability. After the success of the project, Walmart and Dole, Kroger, Nestle, Unilever, and other industry giants cooperated to establish a blockchain technology alliance for supply chain traceability [19]. This study proposes a model for cross-border supply chain management based on the complex computer blockchain for international economic cooperation scenarios, compares and analyzes decision making in two scenarios of unimplemented and implemented blockchain in the cross-border supply chain, and investigates the necessary conditions for implementing blockchain in cross-border supply chain.

## 3. Model Description and Assumptions

In this study, a model for a cross-border supply game with a dominating manufacturer and the following retailer is developed. The manufacturer produces a cross-border product and sells it through a retailer. The decision variables for the manufacturer are the wholesale price *w* and the product cross-border degree *e*, and the decision variable for the retailer is the retail price *p*. When both the manufacturer and the retailer implement a blockchain, the cross-border supply chain can achieve lower transaction costs, build trust, and gain value, while also adding new blockchain application costs. As a result, cross-border goods makers and merchants must consider the benefits and drawbacks before deciding whether or not to deploy blockchain [20].

### 3.1. Cross-Border Supply Chain Costs

Due to information asymmetry and a lack of trust, both producers and retailers face transaction-related search costs, information costs, bargaining costs, and expenses to monitor transaction execution, which are collectively referred to as transaction costs, if blockchain is not deployed. It is assumed that manufacturers and retailers incur equal unit transaction costs. In the case of implementing blockchain, it is assumed that the transaction costs of both the manufacturer and the retailer are fully saved, but both incur blockchain application costs at the same time; without loss of generality, it is assumed that the unit cost of implementing blockchain in the enterprise is greater than the unit transaction cost saved; i.e., *C*_*B*_ > *C*_*T*_. Regardless of whether blockchain is implemented or not, it is assumed that the same production costs exist for manufacturers and the same retail costs exist for retailers [21]. For simplicity, these two types of costs can be considered as zero. Additional cross-border effort costs for the manufacturer to produce the cross-border product can be represented as follows:

(1) $$\begin{array}{c} C\left(e\right)=\frac{1}{2}ke^{2}, \end{array}$$

where *k* is the cross-border effort cost factor.

### 3.2. Cross-Border Product Market Demand

In the case of not implementing blockchain, due to the information asymmetry between enterprises and consumers, consumers cannot accurately and comprehensively grasp the true attributes of cross-border products and the actual cross-border efforts of enterprises, resulting in consumers' inability to fully trust the cross-border degree of products [22]. The negative impact of insufficient consumer trust on the market demand for cross-border products is twofold: first, it weakens the positive impact of product cross-border degree on market demand; second, it directly weakens the potential market size of cross-border products. Therefore, the market demand for cross-border products is assumed to be as follows:

(2) $$\begin{array}{c} D^{N}=a\left(1-\alpha \right)-bp+\beta e\left(1-\gamma \right), \end{array}$$

where *a* is the potential market size of the cross-border product, 0 < *α* < 1 is the potential market size weakening factor of the cross-border product, *b* is the price elasticity coefficient of the cross-border product, *β* shows the cross-border preference degree of consumers, and 0 < *γ* < 1 is the discount factor of the product cross-border degree positively affecting the demand.

In the implementation of the blockchain scenario, consumers fully trust the product cross-border degree, so the cross-border product market demand is transformed as follows:

(3) $$\begin{array}{c} D^{B}=a-bp+\beta e. \end{array}$$

## 4. Cross-Border Supply Chain Decisions in a Blockchain Scenario

The whole life cycle information of cross-border products, especially the cross-border degree information, can be completely and accurately recorded and stored in the product information traceability system supported by blockchain, and consumers can fully trust the cross-border degree of products [23]. Both manufacturers and retailers of cross-border products use the blockchain platform to conduct transactions, and when the number of transactions reaches a certain level, both parties will gain value from the good transaction records. In this scenario, the manufacturer's profit function is computed as follows:

(4) $$\begin{array}{c} \pi_{m}^{B}=\left(w-c_{B}+v\right)D^{B}-\frac{1}{2}ke^{2}. \end{array}$$

The profit function of the retailer can be expressed using the following equation:

(5) $$\begin{array}{c} \pi_{r}^{B}=\left(p-w-c_{B}+v\right)D^{B}. \end{array}$$

As in (4), it can be determined that there is a unique optimal solution for the decision objective function. According to the inverse solution method, the optimal decision result of the manufacturer and retailer is obtained as (5).

The manufacturer's optimal wholesale price can be represented as follows:

(6) $$\begin{array}{c} w^{B^{*}}=\frac{2ak-\left(c_{B}-v\right)\beta^{2}}{4bk-\beta^{2}}. \end{array}$$

In addition, the optimal product cross-border is as follows:

(7) $$\begin{array}{c} e^{B^{*}}=\frac{\beta \left[a-2b\left(c_{B}-v\right)\right]}{4bk-\beta^{2}}. \end{array}$$

Similarly, the optimal profit is computed as follows:

(8) $$\begin{array}{c} \pi_{m}^{B^{*}}=\frac{k{\left[a-2b\left(c_{B}-v\right)\right]}^{2}}{2\left(4bk-\beta^{2}\right)}. \end{array}$$

Likewise, the retailer's optimal retail price is as follows:

(9) $$\begin{array}{c} p^{B^{*}}=\frac{3ak+2\left(c_{B}-v\right)\left(bk-\beta^{2}\right)}{4bk-\beta^{2}}. \end{array}$$

The optimal profit, the market demand in the green supply chain, and the optimal profit can be computed using the following equations, respectively:

(10) $$\begin{array}{c} \pi_{r}^{B^{*}}=\frac{bk^{2}{\left[a-2b\left(c_{B}-v\right)\right]}^{2}}{{\left(4bk-\beta^{2}\right)}^{2}}, \end{array}$$

(11) $$\begin{array}{c} D^{B^{*}}=\frac{bk\left[a-2b\left(c_{B}-v\right)\right]}{4bk-\beta^{2}}, \end{array}$$

(12) $$\begin{array}{c} \pi_{t}^{B^{*}}=\frac{k{\left[a-2b\left(c_{B}-v\right)\right]}^{2}\left(6bk-\beta^{2}\right)}{2{\left(4bk-\beta^{2}\right)}^{2}}. \end{array}$$

The cost of implementing blockchain will negatively affect the product cross-border degree, wholesale price, market demand, and profit of the decision maker. However, the impact on retailers' retail prices depends on the relationship between the product price elasticity coefficient, the degree of consumer cross-border preference, and the cross-border effort cost coefficient and is therefore uncertain. The cost of implementing blockchain has a similar negative effect on the transaction cost of the firm when blockchain is not implemented [24]. Moreover, under the current blockchain technology development and application environment, the cost incurred by enterprises to implement blockchain may be much larger than the transaction cost between enterprises. Therefore, even if enterprises have the appropriate technology, human resources, and other conditions to implement a blockchain, enterprises will face greater cost pressure to implement blockchain. Likewise, the size of the value gain obtained by the enterprise implementing blockchain will also have an important impact on whether the enterprise implements blockchain or not [25].

The relationship between the equilibrium outcome of the game and the unit value gain v obtained by implementing the blockchain in the case of implementing the blockchain is as follows:

(13) $$\begin{array}{c} \frac{\partial e^{B^{*}}}{\partial v}>0\;\frac{\partial w^{B^{*}}}{\partial v}>0,\frac{\partial D^{B^{*}}}{\partial v}>0,\frac{\partial \pi_{m}^{B^{*}}}{\partial v}>0\;\frac{\partial \pi_{r}^{B^{*}}}{\partial v}>0\;\frac{\partial \pi_{t}^{B^{*}}}{\partial v}>0\;\frac{\partial p^{B^{*}}}{\partial v}\left\{\begin{array}{c} >0,bk<\beta^{2}\\ =0,bk=\beta^{2}\\ <0,bk>\beta^{2} \end{array}\right). \end{array}$$

Equation (13) shows that the unit value gain obtained from implementing blockchain positively affects the product cross-border degree, wholesale price, market demand, and profit of the decision maker. For cross-border product manufacturers, the higher the value gain generated by the firm's blockchain implementation, the higher the firm's pricing power of the product, and the easier it is to set high prices. However, the retail price of retailers does not necessarily increase with the increase of value gained from the implementation of blockchain [26]. The impact of the value gain generated by implementing blockchain on retailers' retail prices depends on the relationship between the product price elasticity coefficient, consumer cross-border preference, and cross-border effort cost coefficient.

When *bk* < *β*^2^, the retail price of the retailer increases with the increase of the unit value gain; similarly, when *bk*=*β*^2^, the unit value gain does not affect the retail price of the retailer; and when *bk* > *β*^2^, the retail price of the cross-border product decreases with the increase of the unit value gain. This also means that the increase in value gain resulting from the implementation of blockchain in case *bk* > *β*^2^ not only benefits cross-border supply chain agents but also promotes consumer welfare and social-environmental performance because consumers buy products with a higher cross-border degree at lower prices. It also suggests the possibility of a win-win situation between governments, companies, and consumers. This undoubtedly provides strong evidence of rationality and strong motivation for the “dual-chain integration” of cross-border supply chain and blockchain [27].

## 5. Analysis of Blockchain Implementation Conditions under Different Value Objectives

While using blockchain to minimize transaction costs, boost customer confidence, and generate value for cross-border product makers and merchants, there will be additional blockchain application expenses. The willingness of cross-border supply chains to implement blockchain ultimately depends on the value objectives pursued by cross-border supply chain companies, including environmental value (increased product border crossing) and economic value (increased profits) [28]. Sufficient conditions for implementing blockchain in cross-border supply chains can be analyzed by comparing the product cross-border degree or the profits of manufacturers and retailers before and after implementing blockchain. The following section first examines the requirements for implementing blockchain in cross-border supply chains under both environmental and economic value objectives individually, and then the necessary criteria for attaining both environmental and economic value objectives at the same time. To ensure positive results of each model, the range of values of the potential market size weakening factor for cross-border products is limited to 111. To simplify the expression, it can be represented as

(14) $$\begin{array}{c} \alpha_{2}=\frac{a-2bc_{T}}{a}-\frac{\sqrt{a^{2}{\left[a-2b\left(c_{B}-v\right)\right]}^{2}\left[16b^{2}k^{2}+\beta^{4}{\left(1-\gamma \right)}^{2}-4bk\beta^{2}\left(2-2\gamma +\gamma^{2}\right)\right]}}{a^{2}\left(4bk-\beta^{2}\right)},\\ \alpha_{3}=\frac{2b\left(c_{B}-v\right)\left[4bk-\beta^{2}{\left(1-\gamma \right)}^{2}\right]+a\beta^{2}\gamma \left(\gamma -2\right)}{a\left(4bk-\beta^{2}\right)}-\frac{2bc_{T}}{a},\\ v_{3}=c_{B}+\frac{a\beta^{2}\gamma \left(\gamma -2\right)-2bc_{T}\left(4bk-\beta^{2}\right)}{2b\left[4bk-\beta^{2}{\left(1-\gamma \right)}^{2}\right]},\\ \alpha_{1}=\frac{a-2bc_{T}}{a}-\frac{\left[a-2b\left(c_{B}-v\right)\right]\left[4bk-\beta^{2}{\left(1-\gamma \right)}^{2}\right]}{a\left(1-\gamma \right)\left(4bk-\beta^{2}\right)},\\ v_{1}=\frac{2bc_{n}-a}{2b}+\frac{\left(a-2bc_{r}\right)\left(1-\gamma \right)\left(4bk-\beta^{2}\right)}{2b\left[4b-\beta^{2}{\left(1-\gamma \right)}^{2}\right]}\\ v_{2}=\frac{2bc_{1}-a}{2b}+\frac{\sqrt{b^{2}{\left(a-2bc_{r}\right)}^{2}\left[16b^{2}k^{2}+\beta^{*}{\left(1-\gamma \right)}^{2}-4bk\beta^{2}\left(2-2\gamma +\gamma^{2}\right)\right]}}{2b^{2}\left(4bk-\beta^{2}{\left(1-\gamma \right)}^{2}\right]}. \end{array}$$

**Corollary 1 .**

When (1) v > v_1_ or (2) 0 < v < v_1_ and *α*_1_ < *α* < *a* − 2*bc*_*T*_/*a*, there is *e*^*B*^*∗*^^ > *e*^*N*^*∗*^^; i.e., the product cross-border degree in the case of implementing blockchain in the cross-border supply chain is greater than that in the case of not implementing it.

Corollary 1 gives sufficient conditions for implementing blockchain in cross-border supply chains under the environmental value objective. Increasing the product cross-border degree requires more cross-border effort, which increases the cost of cross-border effort. Therefore, cross-border supply chains need to be given sufficient incentives to increase product cross-border degree; i.e., (i) the unit value gain generated by implementing blockchain is greater than a certain value (higher value gain) or (ii) the unit value gain generated by implementing blockchain is less than a certain value (lower value gain) but the potential market size erosion factor for cross-border products is greater than a certain value (higher degree of market erosion) [29].

## 6. Numerical Analysis

In this section, we use numerical examples to analyze the sufficient conditions for implementing blockchain in cross-border supply chains, the changes in pricing strategies, and the market demand after implementing blockchain in cross-border supply chains under the simultaneous realization of environmental and economic value objectives [30]. Since the size relationship between *bk* and *β*^2^ is not clear, the following is a comparative analysis of the two scenarios of *bk* > *β*^2^ and *bk* < *β*^2^. Meanwhile, to facilitate the comparative analysis of the changes in pricing strategy and market demand after the implementation of blockchain in the cross-border supply chain, the unit value gain *v* is considered as a constant value, and the comparative analysis is conducted from the two cases of high unit value gain (*v*_*H*_ > *c*_*B*_ − *c*_*T*_) and low unit value gain (*v*_*L*_ < *c*_*B*_ − *c*_*T*_). Without loss of generality, the model parameters are assigned as *a* = 500 and *b* = 3.

### 6.1. Analysis of Sufficient Conditions for Implementing Blockchain in Cross-Border Supply Chain

#### 6.1.1. Conditions from the Perspective of Obtaining Higher Unit Value Gain

For implementing blockchain from the perspective of obtaining higher unit value gain for cross-border product manufacturers and retailers under different value objectives, the *v*_*i*_(*i*=1,2,3) is the lower bound threshold of the conditions. A larger *v*_*i*_(*i*=1,2,3) value indicates a higher value gain requirement for cross-border supply chain companies to implement blockchain. Figures 2(a) and 2(b) show that *v*_1_ < *v*_3_ < *v*_2_ < 30. *v* > *v*_1_ areas above 0 < *γ* < 1 range that are split into three blocks by *v*_2_ and *v*_3_. According to Corollary 1, when *v* > *v*_1_, there are *e*^*B*^*∗*^^ > *e*^*N*^*∗*^^; when *v* > *v*_3_, there are *π*_*r*_^*B*^*∗*^^ > *π*_*r*_^*N*^*∗*^^. This means that the implementation of blockchain in cross-border supply chains under the environmental value objective requires the lowest degree of value gain, while the implementation of blockchain for retailers under the economic value objective requires a lower degree of value gain than that for manufacturers.

Comparing Figures 2(a) and 2(b), we find that the size relationship between *bk* and *β*^2^ does not affect the size relationship between *v*_1_, *v*_2_, *v*_3_ but affects the range of their values. Compared with the *bk* > *β*^2^ scenario, the lower threshold value of the unit value gain *v* will become smaller when *bk* < *β*^2^ which means that the value gain condition of the cross-border supply chain implementing blockchain will become lower. The *bk* > *β*^2^ scenario can be interpreted as a larger consumer cross-border preference or a larger impact of cross-border preference. The greater the consumer cross-border preference, the greater the market demand for cross-border products, and the greater the profit earned by manufacturers and retailers, so the value gain condition for implementing blockchain in cross-border supply chains will become more lenient in the *bk* < *β*^2^ scenario. In addition, when *bk* < *β*^2^, the *γ* value corresponding to *v*_1_=0 will become smaller. That is, the lower bound value of the demand discount factor *v* > 0 for the positive impact of product cross-border degree required for manufacturers to be willing to implement blockchain under the environmental value objective will also become smaller as long as the unit value gain is *γ*.

#### 6.1.2. Conditions from the Perspective of Enhancing the Scale of Market Demand for Cross-Border Products

In the case of low unit value gain obtained from implementing blockchain, it is known from the previous inference results that cross-border supply chains under different value objectives have incentives to implement blockchain only when the potential market size weakening factor of cross-border products is greater than a certain degree. This means that the larger the value *α*_*i*_(*i*=1,2,3), the higher the requirement of implementing blockchain for cross-border supply chain companies in terms of weakening the potential market size of cross-border products. Figures 3(a) and 3(b) show the critical values of the potential market size erosion factor for cross-border products under different value objectives. They also show that there is a constant 0 < *α*_1_ < *α*_3_ < *α*_2_ < 0.12 in the range of 0 < *γ* < 1. Similar to Figures 2(a) and 2(b), the area above *α* > *α*_1_ is divided into three blocks by *α*_2_ and *α*_3_.

When the value gain obtained by implementing blockchain is low, the implementation of blockchain in the cross-border supply chain under the environmental value objective requires the lowest degree of weakening of the potential market size for cross-border products, while the implementation of blockchain for the retailer under the economic value objective requires a lower degree of weakening of the potential market size for cross-border products than that for the manufacturer.

Comparing Figures 3(a) and 3(b), we find that the size relationship between *bk* and *β*^2^ also does not affect the size relationship between *α*_1_, *α*_2_, *α*_3_ but affects the range of their values. Compared with the *bk* > *β*^2^ case, the lower threshold value of the potential market size weakening factor *α* for cross-border products will become smaller when *bk* < *β*^2^; i.e., the market demand size increase condition for implementing blockchain in cross-border supply chains will also become lower.

In addition, *γ* values corresponding to *α*_1_=0 and *α*_3_=0 will become smaller when *bk* < *β*^2^.

Figures 4(a) and 4(b) show that if the unit value gain from blockchain implementation is higher, the manufacturer's wholesale price is greater in the case of blockchain implementation than in the case of no blockchain implementation, within the range of values of the demand discount factor.

Figures 5(a) and 5(b) show that if the unit value gain from blockchain implementation is lower (*v*_*L*_=20), the manufacturer's wholesale price is also greater in the case of blockchain implementation than in the case of no blockchain implementation for a range of values of the positive product greenness impact demand discount factor 0 < *γ* < 1 and the potential market size erosion factor 0.12 < *α* < 0.68 for cross-border products.

### 6.2. Analysis of Changes in Retail Prices of Retailers' Characteristics

Figures 6(a) and 6(b) show that if the unit value gained from implementing blockchain is higher, the retail price in the case of implementing blockchain is greater than in the case of not implementing blockchain, within the range of values of the demand discount factor.

Figures 7(a) and 7(b) show that the retail price in the case of blockchain implementation is greater than in the case of no blockchain implementation if the unit value gain due to the implementation of blockchain is lower.

Comparing Figures 6 and 7(a), we find the following: (i) The retailer's retail price in the scenario *bk* > *β*^2^ is less than that in the scenario *bk* > *β*^2^, regardless of whether blockchain is implemented. That is, the higher the degree of consumer's cross-border preference, the higher the retail price set by the retailer. (ii) When *bk* > *β*^2^, the higher the unit value gain from implementing blockchain, the smaller the retail price set by the retailer; when *bk* < *β*^2^, the higher the unit value gain from implementing blockchain, the larger the retail price set by the retailer.

The result of statement (ii) can be interpreted as follows: retailers will pay more blockchain application costs in the case of implementing blockchains in the cross-border supply chain, but consumers' cross-border preference still plays an important role in retailers' pricing decisions. When the consumer's cross-border preference is small, even if the retailer's value gain is increasing, the retailer still needs to set a lower price to attract consumers to buy low-carbon products; on the other hand, when the consumer's cross-border preference is large, there is still enough market demand for the retailer to set a higher price, and the larger the retailer's value gain, the more likely that the retailer sets a higher price.

## 7. Conclusions

The use of blockchain in cross-border supply chains can solve the problem of information asymmetry between enterprises and between enterprises and consumers, lowering transaction costs and increasing supply chain efficiency, as well as increasing consumer trust in cross-border products and increasing market demand for cross-border products. In this study, a game model of the cross-border supply chain is constructed from the perspectives of reducing transaction costs, building trust, and gaining value. Furthermore, the differences in decision outcomes between the non-implementation and implementation of the blockchain are explored and analyzed in cross-border supply chains to determine the sufficient conditions for implementing blockchain in the cross-border supply chain under different value objectives. The main finding under the assumption that cross-border supply chains achieve both environmental and economic value objectives is that both cross-border product manufacturers and retailers have perfect incentives to implement blockchain when the value gain is high, especially when the incremental cost is low. Both cross-border product manufacturers and retailers will increase their selling prices after implementing blockchain. With sufficient conditions for cross-border supply chain companies to be willing to implement blockchain, the cross-border product market demand, product cross-border degree, and optimal profitability for both manufacturers and retailers will improve after implementing blockchain. Future research will explore the conditions for implementing blockchain in cross-border supply chain companies and its corresponding decisions from a dynamic value gain perspective.

## Figures and Tables

**Figure 1:** Cross-border e-commerce supply chain.

**Figure 2:** (a) *bk* > *β*^2^, critical value of unit value gain v. (b) *bk* < *β*^2^, critical value of unit value gain v.

**Figure 3:** *bk* > *β*^2^, critical value of unit value gain *α*.

**Figure 4:** High-price selling relationship under different parameter settings. (a) Wholesale price. (b) Wholesale price at high-value gain at *bk* < *β*^2^.

**Figure 5:** Low-price sales relationship under different parameter settings. (a) Wholesale prices at low-value gain at. (b) Wholesale prices at low-value gain at *bk* < *β*^2^.

**Figure 6:** (a) Retail price at high-value gain at *bk* > *β*^2^. (b) Retail price at high-value gain at *bk* < *β*^2^.

**Figure 7:** Retail price relationship under different parameter settings. (a) The income relationship of retail low prices. (b) The income relationship of retail high prices.

## Data Availability

The data used to support the findings of this study are available from the corresponding author upon request.
